RETRACTED

# Effect of Modified Xianglian Pingwei Powder plus Glutathione and Levofloxacin Hydrochloride on Patients with Liver Cirrhosis and Positive Small Intestinal Bacterial Overgrowth

**DOI:** 10.1155/2022/5063088

**Published:** 2022-04-11

**Authors:** Shanshan Su, Qingqing Wang, Fang Wei, Guoqi Zheng

**Affiliations:** Digestive Department, Cangzhou Central Hospital, Cangzhou, Hebei, China

## Abstract

Liver cirrhosis is a common chronic disease in China. The effect of modified Xianglian Pingwei powder plus Western medicine in the treatment of liver cirrhosis and positive small intestinal bacterial overgrowth is promising. Totally, 100 patients with liver cirrhosis and positive intestinal bacterial overgrowth in Cangzhou Central Hospital from February 2020 to February 2021 were enrolled and randomized via the random number table method at a ratio of 1 : 1 into the study group and control group. The control group received glutathione and levofloxacin hydrochloride, and the study group received Xianglian Pingwei powder plus glutathione and levofloxacin hydrochloride. The traditional Chinese medicine (TCM) syndrome scores, serum aspartate aminotransferase (AST), alanine aminotransferase (ALT), and total bilirubin (TBIL) levels of the two groups were decreased after treatment with lower results in the study group. Xianglian Pingwei powder plus glutathione and levofloxacin hydrochloride was associated with a significantly lower positive rate of small intestine bacterial growth, serum endotoxin level, and peripheral blood toll-like receptor 2 (TLR2) and TRL4 levels versus glutathione and levofloxacin hydrochloride. The combined medication achieved a higher efficacy (90.00%) versus glutathione and levofloxacin hydrochloride (66.00%). The two groups experienced similar safety. Xianglian Pingwei powder plus glutathione and levofloxacin hydrochloride achieved significant benefits of clinical efficacy with a high safety profile in patients with liver cirrhosis versus glutathione and levofloxacin hydrochloride.

## 1. Introduction

Liver cirrhosis is a common chronic progressive liver disease caused by diffuse liver damage from one or more causes with prolonged or repeated action [1]. In China, most cases are posthepatitis cirrhosis and a few are alcoholic cirrhosis and schistosomiasis cirrhosis [2]. Histopathology showed extensive necrosis of liver cells, nodular regeneration of residual liver cells, connective tissue hyperplasia, and fibrous septum formation, which lead to the destruction of hepatic lobule structure and formation of pseudolobule [3]. Consequently, the liver gradually deforms, hardens, and develops into cirrhosis. In the early stage of disease, the strong compensatory function of the liver results in the insidiousness of symptoms [4]. The main manifestations in the later stage include liver function damage and portal hypertension [5], and complications such as upper gastrointestinal bleeding, hepatic encephalopathy, secondary infection, hypersplenism, ascites, and canceration are frequently seen [6].

RETRACTED

Portal hypertension may cause symptoms such as constipation and abdominal distension, resulting in adverse effects on the hepatoenteric circulation and further development of the small intestinal bacteria overgrowth (SIBO) [7]. Research has shown a high prevalence of SIBO in patients with liver cirrhosis [8]. Currently, antibiotics are the mainstay of treatment but are prone to drug resistance. Cirrhosis is a liver dysfunction due to tissue disorders and currently relies on early diagnosis and treatment to control disease progression. Traditional Chinese medicine (TCM) liver preservation therapy is effective in improving clinical symptoms and liver function indicators. Hui et al. [9] pointed out that Xianglian Pingwei powder could effectively relieve the clinical symptoms of patients. Accordingly, this study was conducted to explore the treatment effectiveness of Xianglian Pingwei powder.

## 2. Materials and Methods

### 2.1. General Information

A total of 100 patients with liver cirrhosis and SIBO were randomized into two groups. The study protocol was ethically approved by the Ethics Committee of Cangzhou Central Hospital (2020–344/33).

### 2.2. Inclusion and Exclusion Criteria

Inclusion criteria were as follows: aged ≥18 years old; with different etiologies of chronic liver disease and cirrhosis; and clinical, laboratory, and imaging findings suggest abnormal liver function and/ or portal hypertension and/or histological manifestations of liver cirrhosis [10].

Exclusion criteria were as follows: with various types of infectious bowel diseases; with various types of functional bowel diseases; with intestinal malignancies; and with other primary bowel diseases.

## 3. Methods

### 3.1. Control Group

The patients were given an injection of 0.6 g reduced glutathione (manufacturer: Chongqing Yaoyou Pharmaceutical Co., Ltd.; approval number H20050667) once a day and 0.2 g levofloxacin hydrochloride capsules orally, 3 times a day.

### 3.2. Study Group

In addition to the medication of glutathione and levofloxacin hydrochloride capsules, the patients in the study group were given Xianglian Pingwei powder. The ingredients of Xianglian Pingwei powder include *Magnolia officinalis* 15 g, tangerine peel 15 g, *Atractylodes* 12 g, *Costus* root 10 g, ginger 10 g, jujube 5 g, and roasted licorice 5 g, with one dose administered half in the morning and half in the evening per day. All patients were followed up for 1 month.

RETRACTED

### 3.3. Observation Indicators

1. Assessment of TCM symptom scores includes 9 domains such as nausea and vomiting, anorexia, drowsiness, and fatigue, with each item scored 0–6 points and a total score of 0–36 points. The higher the score, the more severe the symptoms [11].
2. Small intestinal bacterial growth: the lactulose hydrogen breath test was performed with a hydrogen detector (Bedfont, UK). One day before the test, the patients were prohibited from eating spicy and other irritating foods, soy products, milk, and other indigestible foods. The fasting hydrogen concentration on the next day was determined, followed by the intake of 10 g lactulose oral liquid and the assay of hydrogen concentration within 2 hours, once every 15 minutes. A rise in hydrogen concentration above 12 ppm or a fasting hydrogen concentration above 20 ppm after oral administration of lactulose is considered positive.
3. Serum endotoxin level: 1 ml of fasting peripheral venous blood was collected and placed in an anticoagulation tube to determine the endotoxin level using a spectrophotometer (Shanghai Unico) with the chromogenic matrix limulus reagent (Zhanjiang Andus Co., Ltd.).
4. Peripheral blood toll-like receptor 2 (TLR2) and TLR4 levels were determined by flow cytometry (BD FACS Calibur, BD Company, USA).
5. Safety: no adverse reactions were interpreted as level 1 (safe). Mild adverse reactions that allowed for continued medication and did not require special management were interpreted as level 2 (relatively safe). Severe adverse reactions that allowed for continued medication and required special management were as interpreted as level 3 (safety issues). Serious adverse reactions that required discontinuation of medication were considered level 4 (with serious safety issues) [12].
6. Efficacy cured: after treatment, the number of bacteria in the small intestine of the patient is 10^2^–10^5^/ml, without symptoms such as constipation and abdominal distension; markedly effective: after treatment, the patient has significantly fewer bacteria in the small intestine, without symptoms such as constipation and abdominal distension; effective: after treatment, the patient has a small number of bacteria in the small intestine (10^5^/ml and above), with mild symptoms such as constipation and abdominal distension; ineffective: the number of bacteria in the small intestine of the patient continues to increase after treatment, with unrelieved or deteriorated symptoms such as constipation and diarrhea [13].

### 3.4. Statistical Analysis

All data analyses were done by SPSS 21.0. The counting data and measurement data were expressed as rate and (*x* ± *s*) and analyzed using the *χ*^2^ test or rank sum test and *t*-test or *F*-test. A *p* value of 0.05 or lower was claimed as statistical significance.

RETRACTED

## 4. Results

### 4.1. Comparison of General Information

The baseline characteristics of the study group (18 (36.00%) females and 32 (64.00%) males, aged 35–75 years old, and an average age of (55.14 ± 9.35) years, 14 cases (28.00%) with a course of disease of 2–5 years, 36 cases (72.00%) of 6–8 years, 16 cases in grade A (32.00%) and 22 cases in grade B (44.00%), and 12 cases in grade C (24.00%) in terms of Child-Pugh classification) were comparable with those of the control group (19 (38.00%) females and 31 (62.00%) males, aged 36–76 years old, and an average age of (56.02 ± 9.85) years, 15 cases (30.00%) with a course of disease of 2–5 years, 35 cases (70.00%) of 6–8 years, 17 cases in grade A (34.00%) and 20 cases in grade B (40.00%), and 13 cases in grade C (26.00%) in terms of Child-Pugh classification) (*p* > 0.05).

### 4.2. Comparison of TCM Syndrome Scores and Liver Function

The TCM syndrome scores, serum aspartate aminotransferase (AST), alanine aminotransferase (ALT), and total bilirubin (TBIL) levels of the two groups decreased after treatment with lower results in the study group (*p* > 0.05) (Table 1).

### 4.3. Comparison of Small Intestinal Bacterial Growth, Serum Endotoxin Levels, and Peripheral Blood TLR2 and TRL4 Levels

Xianglian Pingwei powder plus glutathione and levofloxacin hydrochloride was associated with a significantly lower positive rate of small intestine bacterial growth, serum endotoxin level, and peripheral blood TLR2 and TRL4 levels versus glutathione and levofloxacin hydrochloride (*p* < 0.05) (Table 2).

### 4.4. Comparison of Clinical Efficacy

The combined medication achieved a higher efficacy (90.00%) versus glutathione and levofloxacin hydrochloride (66.00%) (*Z* = 2.608, *p* < 0.05) (Table 3).

### 4.5. Comparison of Safety

The two groups showed a similar safety profile with comparable incidence of adverse events (*Z* = 0.718, *p* > 0.05) (Table 4).

## 5. Discussion

In the present study, the TCM syndrome scores and serum AST, ALT, and TBIL levels of the two groups decreased after treatment with lower results in the study group, and the combined medication achieved a higher efficacy (90.00%) versus glutathione and levofloxacin hydrochloride (66.00%), which is presumably attributable to the relief of gastrointestinal discomfort symptoms by Xianglian Pingwei powder. Liver cirrhosis is caused by long-term chronic liver damage or repeated increase of liver biochemical indicators, leading to liver inflammation, liver stellate cells activation, and fibrous tissue deposition [14]. The causes of liver cirrhosis include viral hepatitis and chronic viral hepatitis, such as hepatitis B and hepatitis C. In addition, fatty liver is also considered a possible contributory factor, such as inflammatory fatty liver and repeated transaminase elevation, and long-term transaminase elevation without effective treatment may also cause cirrhosis. Therefore, liver cirrhosis is mainly attributed to viral hepatitis, fatty liver, or chronic drug-induced liver injury, autoimmune hepatitis, and other chronic liver damage, which leads to long-term increase in transaminase and subsequent liver cirrhosis. The formation of cirrhosis is divided into compensated and decompensated phases. The treatment for cirrhosis mainly includes antiviral therapy, alcohol withdrawal, effective monitoring, and regular review to prevent complications or space-occupying lesions. Cirrhosis of the decompensated period may induce various complications, such as ascites, pericardial effusion, upper gastrointestinal bleeding, and liver coma, which require effective interventions. In recent years, the incidence of liver cirrhosis has been on arise due to the changes in people's lifestyles. Currently, antibiological drugs such as amoxicillin and levofloxacin hydrochloride capsules are more commonly used in the treatment of patients with liver cirrhosis and SIBO. Nevertheless, long-term antibiotics are predisposed to drug resistance.

RETRACTED

In TCM, constipation and abdominal distension are the main clinical symptoms of patients with liver cirrhosis and SIBO [15], and liver depression and damp-heat of the spleen and stomach are considered the main pathogenesis, which necessitate the regulation of the liver, spleen, and stomach. Among the ingredients of Xianglian Pingwei powder, *Magnolia officinalis* promotes Qi, *Costus* root, Rhizoma Atractylodis, and tangerine peel remove dampness and reinforce the spleen, Chuanlian clears heat and dry dampness, and jujube, ginger, and roasted licorice reconcile the main medicine [16]. The combination of these medicinal herbs can regulate the spleen and stomach, clear heat, and remove dampness. Modern pharmacological research has confirmed [17] that *Magnolia officinalis* can effectively relieve abdominal distension, and *Atractylodes japonicus* and tangerine peel can promote the alleviation of appetite loss. A prior study has shown [18] that in the treatment of patients with liver cirrhosis and SIBO, Western medicine combined with Xianglian Pingwei powder can effectively inhibit the patient's intestinal bacterial overgrowth and yield a good clinical effect. Additionally, it can greatly lower the patient's peripheral blood endotoxin, TLR2, and TLR4 levels.

RETRACTED

It has been reported [19] that bacterial growth involves the release of endotoxins in patients with liver cirrhosis and SIBO, which damages the liver function, resulting in aggravated liver cirrhosis, portal pressure, and stomach intestinal congestion. Furthermore, cytokines such as endotoxin can easily induce the secretion of TRL2 and TLR4. TLR2 and TLR4 mainly identify Gram-positive bacteria and Gram-negative bacteria, respectively, with a strong relation to the severity of the patient's condition. Therefore, TLR2 and TLR4 feature a high application value in the evaluation of clinical efficacy and prognosis of patients. TLR can activate neutrophils, promote the aggravation of inflammatory response [20], identify endotoxins, and conduct inflammatory signals, which are associated with disease aggravation. Notably, the results of the present study showed that Xianglian Pingwei powder plus glutathione and levofloxacin hydrochloride was associated with a significantly lower positive rate of small intestine bacterial growth, serum endotoxin level, and peripheral blood TLR2 and TRL4 levels versus glutathione and levofloxacin hydrochloride. No significant difference was observed in safety between the two groups, indicating that modified Xianglian Pingwei powder plus glutathione and levofloxacin hydrochloride can mitigate the inflammatory reactions in patients, which may be attributed to the inhibition of inflammatory factors by Xianglian Pingwei powder.

## 6. Conclusion

To sum up, Xianglian Pingwei powder plus glutathione and levofloxacin hydrochloride achieved significant benefits of clinical efficacy with a high safety profile in patients with liver cirrhosis versus glutathione and levofloxacin hydrochloride.

## Figures and Tables

**Table 1:** Comparison of TCM syndrome scores and liver function ($\bar{x}\pm s$).

Groups	*n*	Time	TCM syndrome (points)	AST (U/L)	ALT (U/L)	TBIL (*μ*mol/L)
Study group	50	Before medication	18.64±3.68	101.63±9.80	174.38±9.16	35.35±5.97
		After medication	8.56±1.52	42.28±7.47	49.88±7.44	19.05±3.76
Control group	50	Before medication	18.82±3.03	97.96±9.38	119.51±9.36	36.31±6.65
		After medication	15.02±2.10	52.85±8.94	68.16±9.32	29.47±5.28

AST, aspartate aminotransferase; ALT, alanine aminotransferase; TBIL, total bilirubin.

**Table 2:** Comparison of small intestinal bacterial growth, serum endotoxin levels, and peripheral blood TLR2 and TRL4 levels ($\bar{x}\pm s$).

Groups	*n*	Time	Positive bacterial growth in the small intestine	Endotoxin (EU/ml)	TLR2 (GMF)	TRL4 (GMF)
Study group	50	Before medication	50 (100.00)	0.33 ±0.08	80.28 ±8.93	30.06 ±5.18
		After medication	9 (18.00)	0.06 ±0.02	35.88 ±5.06	11.06 ±1.48
Control group	50	Before medication	50 (100.00)	0.31 ±0.10	79.88 ±9.00	29.96 ±5.03
		After medication	21 (42.00)	0.13 ±0.06	50.18 ±9.13	19.40 ±4.18

RETRACTED

**Table 3:** Comparison of clinical efficacy (*n* (%)).

Groups	*n*	Cured	Markedly effective	Effective	Ineffective	Total effectiveness
Study group	50	3 (6.00)	16 (32.00)	26 (52.00)	5 (10.00)	45 (90.00)
Control group	50	1 (2.00)	11 (22.00)	21 (42.00)	17 (34.00)	33 (66.00)
*Z*						2.608
*P*						0.009

**Table 4:** Safety comparison (*n* (%)).

Groups	*n*	Level 1	Level 2	Level 3	Level 4
Study group	50	45 (90.00)	2 (4.00)	2 (4.00)	1 (2.00)
Control group	50	47 (94.00)	1 (2.00)	1 (2.00)	1 (2.00)
*Z*					0.718
*P*					0.473

## Data Availability

The datasets used to support the findings of this study are available from the corresponding author upon request.
